# Point-of-Care Cardiac Ultrasound Training Programme: Experience from the University Hospital Hradec Králové

**DOI:** 10.1155/2024/9974284

**Published:** 2024-01-06

**Authors:** Petr Grenar, Jiří Nový, Karel Mědílek, Martin Jakl

**Affiliations:** ^1^Department of Emergency Medicine, University Hospital Hradec Králové, Hradec Králové, Czech Republic; ^2^First Department of Cardio-Angiology and Internal Medicine, University Hospital Hradec Králové, Hradec Králové, Czech Republic; ^3^Department of Military Internal Medicine and Military Hygiene, Faculty of Military Health Sciences, University of Defence, Hradec Králové, Czech Republic

## Abstract

Point-of-care ultrasound examinations performed by physicians of different specialties are a rapidly growing phenomenon, which has led to a worldwide effort to create a standardised approach to ultrasound examination training. The implementation of emergency echocardiography by noncardiologists is mainly aimed at the standardisation of the procedure, a structured training system, and an agreement on competencies. This article summarises the current training programmes for nonechocardiographers at the University Hospital in Hradec Králové. In cooperation with cardiologists specialised in cardiac ultrasound (ECHO), an extended acute echo protocol dedicated to emergency department physicians was developed and validated in daily practice. According to our retrospective evaluation, after one year of clinical practice, we can confirm that point-of-care ultrasound examinations performed using the standardised limited echo protocol are safe and accurate. The observed concordance with comprehensive ECHO was 78%. This trial is registered with NCT05306730.

## 1. Introduction

Point-of-care ultrasonography (POCUS) is defined as the acquisition, interpretation, and immediate clinical integration of ultrasonographic imaging performed by acute care clinicians at the patient's bedside rather than by a radiologist or cardiologist [1, 2]. With the increasing quality and availability of ultrasound equipment, POCUS is being more widely performed by a variety of specialists [3]. Despite the growth in the importance and presumed benefits of POCUS, there is no comprehensive and generally accepted consensus on the required level of investigation at the time of writing this article [1, 4–20]. The absence of a training programme and the introduction of this diagnostic method without clearly defined examination protocols and rules for its use led the Joint Commission on Accreditation of Healthcare Organizations and the Emergency Care Research Institute to identify the adoption of POCUS as a major health technology hazard in 2020 [21]. In the same year, a statement on the need for structured educational programmes for POCUS was published by the Ultrasound Working Group of the European Federation of Internal Medicine [22]. Additionally, in 2020, the American Society of Echocardiography stated that to ensure high-quality care, cardiologists should be involved in the education and direct training of clinicians who perform cardiac ultrasonography [23]. With reference to Dr. Kimura's original work, the different levels of cardiac ultrasound examination are described according to the extent of the examination [23, 24]. The definition of these terms is essential to define a universal POCUS training programme for use across different specialties (internal medicine, emergency medicine, intensive care, anaesthesia, etc.). Cardiac ultrasound categories are shown in Table 1. The findings of cardiac POCUS should always be evaluated in the context of a comprehensive examination with the awareness of the potential for misinterpretation in view of the known limitations of this method (time constraints, limited patient examinability, examiner experience, etc.) [12, 19, 25, 26]. In 2013, the European Association of Cardiovascular Imaging (EACVI) recommended following the ABCD approach when performing emergency echocardiography, which is shown in Table 2 [25, 27].

## 2. Cardiac POCUS Training Programme in the University Hospital Hradec Králové

In 2020, on the initiative of the physicians of the First Internal Cardiology Clinic and the physicians of the Emergency Medicine Department, a pilot training programme for limited echocardiography was launched for physicians without cardiology qualifications. The British Society of Echocardiography (BSE) Level 1 protocol was chosen as the echocardiography training scope, extended by apical two- and three-chamber views and measurement of the tricuspid valve gradient for pulmonary hypertension estimation and the ascending aortic dimension. Color Doppler of the aortic and mitral valves from parasternal long and short axis views and the mitral valve from apical views was also added. This protocol was chosen to cover major abnormalities of the right and left ventricles and aortic, mitral, and tricuspid valves to assess pulmonary hypertension and pericardial effusion. It may also raise suspicion of a dissection of the ascending aorta. The protocol also includes a lung ultrasound (see Figure 1) [28] to assess the most significant pulmonary diseases. The ultrasound training programme consists of the following steps.

### 2.1. Step One: Basic Echocardiography Introduction—Theoretical Course

Physicians who had not previously received systematic training in any form of ultrasonography were offered participation in the training programme.

A three-hour introductory seminar is provided to introduce students to the principles of focused ultrasound examination and the required echocardiography protocol. The theoretical training includes a presentation of possible pathological findings on lung ultrasound and their place in the overall examination protocol. For theoretical preparation, a basic textbook on echocardiography is recommended (e.g., Echo Made Easy or Point of Care Ultrasound [29, 30]).

Following the introduction, trainees under the guidance of a cardiologist learn how to operate the ultrasound machine to optimise the projection display and archive individual recordings.

### 2.2. Step Two: Training in Clinical Practice

The actual clinical training takes place at the Department of Emergency Medicine and the Department of Noninvasive Cardiology of the First Department of Internal Medicine. Under the supervision of trainers, who are board-certified cardiologists with many years of experience in echocardiography, trainees perform an ultrasound examination of the heart according to a defined protocol. Individual digital images are archived in a central repository. A structured record of each examination is stored in the hospital information system.

The duration of this phase can vary, and it is necessary for trainees to become familiar with the most common pathologies required for the logbook. The minimum period of clinical training is three months.

### 2.3. Step Three: The Final Assessment

The formal examination takes place in the presence of two cardiologists with extensive echocardiography experience, one holding EACVI accreditation in adult transthoracic echocardiography and the other being proficient in emergency medicine.

The examination consists of an independently performed echocardiographic examination as per protocol under the supervision of examiners who assess the quality and completeness of the study. The candidate makes a report based on acquired images, which is scrutinised for accuracy and guidance for the next management of the patient. In the second part, the candidate is presented with a randomly selected echo study based on the protocol. Correct interpretation of the findings is marked.

In the case of a positive evaluation by both examiners, the trainees receive a certificate on the successful completion of the course. Based on this, the candidates' personal work competencies are extended by independently performing and reporting on emergency cardiac ultrasound examinations.

To maintain examination quality and competence, a minimum of fifty examinations per year must be documented, and once per year, a four-hour stay at the echo department under the supervision of the supervisor is required to formally verify the maintenance of examination quality. All examinations must be recorded in the hospital information system.

## 3. Effectiveness of the Training Programme: Experience after One Year of Practice

In 2022, a total of 560 patients were examined in the emergency department using the limited echocardiography protocol by a noncardiologist who had successfully completed the training programme. Of these, 111 were admitted to the hospital. Full echocardiography examination was recommended by the physician performing the basic echo study in all cases and performed in 69 (62%) of the patients. In this group, the results of both scans were compared with the focus on left and right ventricle dimensions, left ventricle global and regional function, ascending aorta dimension, pulmonary hypertension, significant valvular abnormality and assessment of pericardial space, and inferior vena cava dimension assessment. The study was approved by the local ethics committee. The main focus was the revelation of unrecognised aortic dilatation, unrecognised or misrecognised significant left ventricular dysfunction (left ventricle ejection fraction <40% or focal akinesis), right ventricular dilatation, pulmonary hypertension, significant valvular regurgitation, incorrect assessment of the pericardium and inferior vena cava, or any other missed significant findings resulting in incorrect clinical management. The comparison was limited by the fact that the mean time difference between basic and comprehensive echo studies was 4.2 days (median 2 days), and the clinical status of some patients varied by hours. We can, however, conclude in retrospect that concordance was found for 78% of the patients examined. In 15 cases (the remaining 22%), a discrepancy was found (1 case of overestimated aorta dimension, 2 cases of overestimated LV function, 1 case of underestimated LV function, 1 case of undescribed PK dilatation, 3 cases of undescribed pulmonary hypertension, 1 case of overestimated and 1 case of underestimated valvular lesion, 1 case of undescribed tricuspid annuloplasty ring, 1 case of suspected LV thrombus that was not confirmed, and 1 case of an undescribed regional wall motion abnormality). Of note, none of these discrepancies would have changed or influenced the therapeutic management of the patients.

## 4. Discussion

POCUS is not defined by the scope of the examination but by the conditions under which the examination is performed and the level of expertise of the examining physician. We believe that it is good practice to teach cardiac POCUS to physicians with a wider range of specialties to ensure safe and confident use of this examination method in clinical practice. The scope of the actual examination must always be adapted to the clinical condition of the patient; this is the essence of POCUS. Compared to the established multiday courses for POCUS, the limited echocardiography training programme at the University Hospital Hradec Králové is time-consuming and requires the accessibility of the echocardiography department facilities and the availability of specialist physicians to consult with the candidate regarding their ultrasound findings.

### 4.1. Limitation of the Analysis

The main limitation of this analysis is the fact that the analysed subgroup consisted only of hospitalised patients. This may have led to underestimating errors in patients who were discharged due to an unrecognised echocardiographic finding. This limitation will be addressed by the ENDEMIC study. Another limitation is the delay of the supervision examination (4.2 days), during which some findings could have spontaneously resolved (transient systolic dysfunction, etc.).

## 5. Conclusion

Our experience confirms that the concept of sonography training enables physicians of different specialties to perform standardised ultrasound examinations that, according to our retrospective evaluation, are accurate and reproducible and meet the requirements for safe use according to the ABCD approach. However, high accuracy alone does not justify the cost of a training programme, and there is currently little to no evidence of the clinical benefit of POCUS echocardiography by noncardiologists. To overcome this lack of evidence in patients with chest pain, the prospective, randomised ENDEMIC trial (NCT05306730) was initiated. Publication of the study results is anticipated in mid-2024.

## Figures and Tables

**Figure 1:** Limited ECHO protocol.

**Table 1:** Cardiac ultrasound categories.

Point-of-care ultrasound				Consultative ultrasound	
	UAPE	FOCUS	CCE	Limited ECHO	Comprehensive ECHO
Diagnostic expectations	“US stethoscope” used to augment bedside examination	Focused exams with specific imaging protocols based upon suspicion of specific disease	Focused on a collection of specific views/findings pertinent to the care of the critically ill (e.g., cardiac output, fluid response)	Limited imaging protocol applied to answer a specific question	Comprehensive, all findings, use advanced technics
Quantification	Usually absent	Optional	Typically	Typically	Mandatory
Documentation	Not recorded	Images archived, formal report	Images archived, formal report	Images archived on PACS, formal report	Images archived on PACS, formal report
Teaching required	Weeks	Weeks to months	Months	Months to years	Years

CCE, critical care echocardiography; POCUS, point-of-care ultrasound; UAPE, ultrasound-assisted physical examination; FOCUS, focused cardiac ultrasound. Source: Kimura BJ. Point-of-care cardiac ultrasound techniques in the physical examination: better at the bedside. Heart 2017; 103: 987–994.

**Table 2:** ABCD approach.

(A) Awareness	Avoiding routine
(B) Be suspicious	Verification of ultrasound findings in the context of clinical and other paraclinical investigations
(C) Comprehensiveness	Do as complete examination as suitable
(D) Double R—record, review	The study should be recorded and reviewed

Source: Neskovic AN, Hagendorff A, Lancellotti P, et al. Emergency echocardiography: the European Association of Cardiovascular Imaging recommendations. Eur Heart J Cardiovasc Imaging. 2013; 14 (1): 1–11.

## Data Availability

Dataset is available from the corresponding author upon reasonable request.

## Abbreviations

A2CH: Apical two-chamber view
A3CH: Apical three-chamber view
A4CH: Apical four-chamber view
A5CH: Apical five-chamber view
BSE: British Society of Echocardiography
CCE: Critical care echocardiography
FOCUS: Focused cardiac ultrasound
POCUS: Point-of-care ultrasound
PLAX: Parasternal long axis
SAX: Parasternal short axis
S4CH: Subcostal four-chamber view
UAPE: Ultrasound-assisted physical examination.
